RETRACTED

# Research Status of Differentially Expressed Noncoding RNAs in Type 2 Diabetes Patients

**DOI:** 10.1155/2020/3816056

**Published:** 2020-11-13

**Authors:** Rou Shi, Yingjian Chen, Yuanjun Liao, Rang Li, Chunwen Lin, Liangchang Xiu, Haibing Yu, Yuanlin Ding

**Affiliations:** ^1^Department of Epidemiology and Medical Statistics, Guangdong Medical University, Dongguan, Guangdong 523808, China; ^2^Huizhou Central People's Hospital, Department of Endocrinology, Huizhou, Guangdong 516008, China; ^3^Institute of Medical Systems Biology, Guangdong Medical University, Dongguan, Guangdong 523808, China

## Abstract

Aims. Noncoding RNAs (ncRNAs) play an important role in the occurrence and development of type 2 diabetes mellitus (T2DM). This paper summarized the current evidences of the involvement microRNAs, long noncoding RNAs (lncRNAs), and circular RNAs (circRNAs) in the differential expressions and their interaction with each other in T2DM. Methods. The differentially expressed miRNAs, lncRNAs, and circRNAs in the blood circulation (plasma, serum, whole blood, and peripheral blood mononuclear cells) of patients with T2DM were found in PubMed, GCBI, and other databases. The interactions between ncRNAs were predicted based on the MiRWalk and the DIANA Tools databases. The indirect and direct target genes of lncRNAs and circRNAs were predicted based on the starBase V2.0, DIANA Tools, and LncRNA-Target databases. Then, GO and KEGG analysis on all miRNA, lncRNA, and circRNA target genes was performed using the mirPath and Cluster Profile software package in R language. The lncRNA–miRNA and circRNA–miRNA interaction diagram was constructed with Cytoscape. The aim of this investigation was to construct a mechanism diagram of lncRNA involved in the regulation of target genes on insulin signaling pathways and AGE–RAGE signaling pathways of diabetic complications. Results. A total of 317 RNAs, 283 miRNAs, and 20 lncRNAs and circRNAs were found in the circulation of T2DM. Dysregulated microRNAs and lncRNAs were found to be involved in signals related to metabolic disturbances, insulin signaling, and AGE–RAGE signaling in T2DM. In addition, lncRNAs participate in the regulation of key genes in the insulin signaling and AGE–RAGE signaling pathways through microRNAs, which leads to insulin resistance and diabetic vascular complications. Conclusion. Noncoding RNAs participate in the occurrence and development of type 2 diabetes and lead to its vascular complications by regulating different signaling pathways.

## 1. Introduction

Epidemiological investigation showed that there are approximately 422 million diabetes patients worldwide at present, which is estimated to rise up to 642 million in the global population by 2040 [1]. Among them, more than 90% are with type 2 diabetes mellitus (T2DM), and the trend has been toward a younger population lately [2]. The current trends have made its prevention necessary. Genes and lifestyle could both trigger T2DM with hyperglycemia [3]. Serious complications, such as diabetic, cardiovascular, and cerebrovascular diseases, and diabetic retinopathy, which are the main reasons for deaths among T2DM patients, can be caused by uncontrolled hyperglycemia and could increase the risk of cancer [4–7]. The prevention and treatment of diabetes is a long-term challenge.

RETRACTED

Most studies on type 2 diabetes only focus on 2% of the coding genes (DNAs) and neglect the role of ncRNAs [8]. The deregulation of activity of miRNAs, lncRNAs, and circRNAs in the circulation (peripheral monocytes, whole blood, plasma, and serum) of patients with metabolic and diabetic diseases has been observed [9]. A total of 10,213 experimentally verified human microRNA-lncRNA pairs are included in the StarBase v2.0 database (http://starbase.sysu.edu.cn/starbase2/index.php), but few interaction networks are related to T2DM [10]. Ongoing research on the activity of ncRNAs in the pathogenesis of T2DM provides evidence for the discovery, diagnosis, and management of diabetes.

There is significant evidence, and multiple studies have demonstrated that noncoding RNAs are involved in T2DM regulation and its complications. The altered activity and complex interactions of miRNAs, lncRNAs, and 14 circRNAs in blood tissues were found to be associated with T2DM complications [11–14]. We reviewed and analyzed the data from 85 relevant studies of the two kinds of ncRNAs in T2DM and performed GO and KEGG analyses. Mechanism maps were constructed for three differentially expressed ncRNAs. The regulatory networks of three differentially expressed types of lncRNA–miRNA in T2DM were constructed, and the lncRNA regulatory mechanism maps were constructed based on the insulin signaling pathways and the AGE–RAGE signaling pathways. We used text mining and bioinformatics methods to search for ncRNAs, which are involved in the regulation of T2DM, and predict their targets. Downstream analyses of gene ontology, pathways, and regulatory networks suggested that the insulin signaling pathway, insulin resistance signal transduction, and AGE–RAGE signal transduction are regulated by several ncRNAs. This study provides new evidence and resources regarding ncRNAs which are involved in T2DM regulation. Moreover, these candidate ncRNAs can be used as biomarkers for the diagnosis and detection of diabetes.

## 2. Material and Methods

### 2.1. Search Strategy and Eligible Studies

A total of six databases (PubMed, Google Scholar, Cochrane Library, Wanfang, Weipu, and CNKI) were searched in this investigation. “miRNA” or “microRNA” and “diabetes” or “type 2 diabetes”; “lncRNA” or “long non-coding RNA” and “diabetes” or “hyperglycemias”; “circular RNA” or “circRNA” and “diabetes” or “hyperglycemia” were used as the keywords for search, and it included all studies published before November 30, 2019.

RETRACTED

### 2.2. Study Screening Criteria

Eligible studies were original investigations on ncRNA expression profiles in T2DM patients compared to healthy controls, involving human tissue samples, and published in Chinese or English. We excluded meta-analyses, reports, conference abstracts, abstracts, news, reviews, letters to the editor and editorials, duplicate publications, comparisons of T2DM patients with different complications, studies without normal healthy control samples, those lacking statistically significant differences, and investigations that did not include human data, cell cultures, or animal models (Figure 1).

### 2.3. Data Extraction

Two reviewers extracted data from standard-compliant studies. Tables 1 and 2 show the source of cases, sample sizes of the case group and control group, and statistically significant differences in the ncRNA expression of the selected studies.

### 2.4. Quality Assessment

According to our investigation purpose, the QUADAS2 standard was used to design related questions. The questions in the scale are designed, and a preliminary evaluation is conducted on a few literatures. If the agreement is good, the tool can be used to rate all the included studies; if the agreement is poor, further refinement may be needed. Furthermore, the QUADAS2 scale was used to assess study quality, where ≥8 was considered as excellent, 4~7 was medium, and ≤4 was poor.

### 2.5. Noncoding RNA Target Gene Prediction and Bioinformatics Analysis

lncRNA–miRNA and circRNA–miRNA interactions were predicted with miRWalk and CircInteractome. Cytoscape was used to construct lncRNA–miRNA interactions. The functional relationships of miRNA and lncRNA–miRNA interactions in T2DM were predicted using the DIANA Tools.

Target prediction algorithms experimentally verified codes and databases of miRNA targets on ncRNAs, and the software that can identify potentially altered molecular pathways by expressing single or multiple miRNAs are included in the tool library of the DIANA Tools. Pathway analyses were conducted using the R statistics cluster profiler package (https://www.rdocumentation.org/packages/clusterProfiler/versions/3.0.4) to characterize the functional involvement of putative genes.

## 3. Results

### 3.1. Study Characteristics

Figure 1 shows the document screening and data extraction procedures. A total of 9,923 articles were retrieved in a search of several online databases, and 4,179 remaining articles resulted from a screening of the Materials and Methods to eliminate duplicates, 2,549 of which were not relevant. We excluded reviews, meta-analyses, reports, summaries (*n* = 963), letters to the editor, news and comments, editorials, conference reports (*n* = 649), articles not in English or Chinese (*n* = 18), studies not involving humans (*n* = 377), T1DM (*n* = 28), gestational diabetes studies (*n* = 82), and articles lacking survival data (*n* = 8). The remaining 85 published studies, including a total of 5,914 T2DM patients and 5,682 healthy controls, were selected for analysis.

RETRACTED

Tables 1, 2, and 3 show the study characteristics and data included in the analysis, specific sample size and type, age, sex ratio, RNA trend, and experimental validation methods. All 85 articles reported original investigations. There were 71 studies on miRNA, 9 on lncRNA, and 5 on circRNA among T2DM patients. The 317 dysregulated ncRNAs included 283 miRNAs, 20 lncRNAs, and 14 circRNAs (Tables 1, 2, and 3) identified in the blood tissues. The list of miRNAs was updated with the latest names provided by the miRBase (http://www.mirbase.org), and the lncRNA names were updated with those in the Human Gene Nomenclature Committee prior to analysis.

### 3.2. Quality Assessment

All were of medium or high quality (Tables 1, 2, and 3). Standards 12 and 13 of the QUADOMICS tool did not apply, since none were blinded studies in which the investigators were not aware of the reference standards and patient samples.

### 3.3. GO and KEGG Analysis of miRNA Dysregulation in T2DM

The first three items of GO are transcription factor activity, RNA polymerase II proximal promoter sequence-specific DNA binding (GO: 0000982), posterior synapse (GO: 0098794), and posterior synapse and asymmetric synapse (GO: 0032279), according to *P* < 0.001. The KEGG results reveal many ways for the development of T2DM and its complications. cGMP-PKG, cAMP, MAPK, mTOR, FoxO, TGF-*β*, PI3K-Akt, and Wnt are among the signal transduction pathways involved in energy metabolism. Insulin-related pathways include insulin resistance, insulin signaling, insulin secretion, and pancreatic secretion. Thyroid hormone secretion; parathyroid hormone synthesis, secretion, and function; aldosterone synthesis and secretion; renin secretion of thyroid hormone signaling pathway; endocrine and other factors that regulate calcium absorption; and cell aging and cancer-related pathways are some of the other endocrine-related signaling pathways. At present, the signaling pathway, namely, the AGE–RAGE signaling pathway, is closely related to diabetes complications. A total of 78 signal pathways were identified according to *P* < 0.05, of which the top 20 signal pathways are listed in Figure 2. The AGE–RAGE signaling in diabetic complications, insulin signaling pathway, and insulin resistance were the three pathways used to construct a mechanism diagram (Supplementary Figure 1). The gene expression in the red box is affected by ncRNAs.

RETRACTED

In Figure 2, the vertical axis represents the different signaling path names, and the horizontal axis represents the number of genes enriched in the pathway. The different colors are determined by the *P* value.

### 3.4. GO and KEGG Analysis of lncRNA Dysregulation in T2DM

According to literature extraction and bioinformatics prediction, 10 lncRNAs interacted with 743 microRNAs. A total of 283 miRNAs verified by RT-qPCR were extracted from the literature, of which 41 miRNAs were obtained from the literature and the database. Supplementary Figure 3 shows how an interaction network consisting of 10 lncRNAs and 60 miRNAs was constructed, according to connectivity ≥ 3. lncRNA is shown as a triangle, and miRNA is shown as a square, where red indicates high expression and green indicates low expression. And the predicted miRNA–mRNA interaction is represented by light gray lines.

The first three items of GO are transcription factor activity, RNA polymerase II proximal promoter sequence-specific DNA binding (GO: 0000982), posterior synapse (GO: 0098794), and asymmetric synapses (GO: 0000978), according to *P* < 0.001. The KEGG signaling pathway related to T2DM and its complications are signaling pathways, including cGMP-PKG, mTOR, MAPK, cAMP, AMPK, TGF-beta, and PI3K-Akt.  Figure 3 shows insulin resistance in diabetic complications, AGE–RAGE signaling, and signaling pathways associated with endocrine diseases, including thyroid hormone signaling. A total of 69 signal pathways were identified based on *P* < 0.05. Furthermore, a mechanism diagram was constructed with three signal pathways: AGE–RAGE signal transduction, insulin signal transduction pathway, and the insulin resistance signal (Supplementary Figure 2). The genes shown in red were affected by lncRNAs.

In Figure 3, the vertical axis represents the different signaling path names, the horizontal axis represents the number of genes enriched in the pathway, and the different colors are determined by the *P* value.

### 3.5. GO and KEGG Analysis of the circRNA Dysregulation in T2DM

The first three items of GO are transcription factor activity and RNA polymerase II proximal promoter sequence-specific DNA binding (GO: 0000982), posterior synapse (GO: 0098794), and synaptic membrane (GO: 0097060), according to *P* < 0.001. Signaling pathways related to metabolism, PI3K–Akt, FoxO, MAPK, TGF-beta, and AMPK, and axon guidance and signaling pathways related to endocrine, were included in the KEGG results (Figure 4).

RETRACTED

In Figure 4, the vertical axis represents the different signaling path names, the horizontal axis represents the number of genes enriched in the pathway, and the different colors are determined by the *P* value.

### 3.6. lncRNA-circRNA–miRNA Interaction Network

Figure 5 shows how we constructed an interaction network to illustrate the relationship between three dysregulated ncRNAs in T2DM. The network includes 10 lncRNAs (triangles), 4 circRNAs (circles), and 91 miRNAs (squares), according to connectivity ≥ 3. Among them, 10 lncRNAs and 60 miRNAs have interaction. Furthermore, the interaction of 4 circRNAs and 31 microRNAs, and the miRNA–mRNA interaction are shown as a light gray line. The miRNAs predicted by bioinformatics are light blue, red represents the increase in PCR-validated circulation among T2DM patients, and green represents the decrease in PCR-validated circulation among T2DM patients. It is interesting that both lncRNA (MALAT1, LINC02402) and two circRNAs (cir-0068087 and cir-0054633) interact with two miRNAs (miR-1033 and miR-217).

### 3.7. Perturbed Pathways Mediated by Dysregulated lncRNA–miRNA

Insulin signal dysregulation is the root cause of T2DM and its complications. This study found that eight lncRNAs can participate in insulin signal transduction by regulating 17 miRNAs (Figure 6). The AGE–RAGE signaling pathway is currently the only signaling mechanism believed to cause T2DM complications, including diabetic microvascular and macrovascular lesions. A total of eight lncRNAs can participate in the transduction of AGE–RAGE signal by regulating 12 miRNAs in this investigation (Figure 7).

Figure 6 shows the possible regulatory mechanism of differentially expressed lncRNA–miRNA in the circulation based on the insulin signaling pathway in T2DM.

Figure 7 shows the possible regulation mechanism of lncRNA–miRNA differentially expressed in the circulation based on the AGE–RAGE signaling pathway in T2DM.

## 4. Discussion

Insulin resistance and hyperglycemia are the main features of T2DM as a metabolic disease. Insulin resistance impairs the islet function, and the disease will develop from prediabetes to diabetes when the islets can no longer compensate for insulin resistance. Increasing evidence shows that ncRNAs in the circulation of T2DM patients can be used as biomarkers for the diagnosis and detection of diabetes and its complications [28, 66, 73, 75].

RETRACTED

Significant evidence shows that miRNAs are involved in the regulation of T2DM and its complications [45, 76–78]. This study found that 72 miRNAs are involved in the insulin signaling pathway, 61 are involved in insulin resistance signal transduction, and 61 are involved in the AGE–RAGE signal transduction. miR-495-3p regulates six target genes active in insulin signaling pathways, including GSK-3B, IRS-1, PPP1CB, PRKAA2, PRKAG2, and SOCS3. miR-27a-3p, miR-27b-3p, miR-495-3p, and miR-7-5p interact with IRS1 to affect insulin resistance. Let-7f-5p, miR-4778-5p, miR-7-5p, and miR-92a-3P interact with IRS2 to affect insulin resistance.

The nine lncRNAs dysregulated in T2DM include MEG3, MALAT1, GAS5, CARMEN, lncRNA-MIR503HG, LINC00523, LINCTPV, LINC02402, and lncRNA-MIAT. These ncRNAs target 33 genes that affect insulin resistance (e.g., FOXO1, GSK3B, IRS1/2, and STAT3). Eight lncRNAs (MEG3, MALAT1, GAS5, CARMEN, MIR503HG, LINC02402, PVT1, and MIAT) jointly target 20 genes (such as COL1A2, EDN1, FOXO1, PLCB1, PRKCD, and VEGFC, among others) to participate in the AGE–RAGE signaling. MIAT and MEG3 interact with IRS1/2, and IRS phosphorylation, in turn, affects IRS degradation and insulin resistance. Three types of lncRNA (MEG3, MALAT1, and GAS5) interact with PI3K through the AGE–RAGE signaling, thereby affecting IRS degradation and insulin resistance in T2DM. Both MEG3 and MALAT1 interact with endothelin 1 (EDN1), thus affecting vascular function and leading to diabetic vascular complications. MIAT also interacts with VEGFC, leading to vascular dysfunction.

There is much evidence that lncRNAs can be used as a miRNA sponge to regulate downstream genes and affect the occurrence of various diseases [79–82]. At present, it is believed that the main cause of insulin resistance is the increase of inflammatory cytokines. This interferes with the normal phosphorylation of IRS in insulin signal transduction and blocks a series of cascaded amplification reactions activated by downstream signals, thereby affecting the physiology of insulin production and transport function, causing insulin resistance [83]. Studies have shown that MEG3 protects cardiomyocytes from apoptosis induced by ischemia-reperfusion through the miR-7-5p/PARP1 pathway, which may be a new target for the treatment of myocardial ischemia-reperfusion injury [84]. Studies have also shown that the MEG3/miR-7-5p/EGFR axis is essential for regulating cardiomyocyte autophagy [85]. We also predicted that MEG3/miR-7-5p participates in the metabolism of insulin signals through IRS or activation of MAPK signals (Figure 6), thereby affecting normal insulin signal transduction, leading to the occurrence of insulin resistance and T2DM. However, our prediction results still need much *in vivo* and *in vitro* data to support it. lncRNA GAS5, MEG3, PVT1, and MALATI can be used as sponges to regulate six miRNAs (miR-7-5p, miR-3127-3p, miR-153-5p, miR-96a-5p, miR-495-3p, and let-7-5p). They participate in the activation of the MAPK signal, leading to increased downstream lipid production and induced insulin resistance.

RETRACTED

Most patients with T2DM died of diabetic complications, including vascular complications and microvascular complications. The combination of AGE and RAGE activates downstream NF-*κ*B signaling, leading to an increased expression of adhesins, endothelins, and procoagulant factors, resulting in vascular dysfunction and vascular remodeling [86–88]. PLC and PKC are the key molecules in the AGE–RAGE signaling to activate NF-*κ*B signaling. Long-chain non-coding RNA, GAS5, MEG3, MALAT1, CARMEN, MIR503HG, and LNC02402 can be used as sponge-regulated miRNAs to target two key downstream genes (PLC and PKC), leading to the biological effects of downstream NF-*κ*B signal activation (Figure 7). This is also a key factor in the development of T2DM and its vascular complications. Yue et al. found that the downregulation of GAS5 alleviates palmitic acid-induced myocardial inflammatory injury through the miR-26a/HMGB1/NF-*κ*B axis [89]. The results of Liang et al. showed that GAS5 knockdown restores oxidized low-density lipoprotein-induced impaired autophagy flux via upregulating the miR-26a in human endothelial cells [90]. These findings suggest that GAS5 can act as a sponge for miR-26a to cause inflammation and endothelium cell damage. Our investigation speculates that GAS5 can interact with miR-26a, target PLC and PKC, activate NF-*κ*B, and cause inflammation and damage to the vascular endothelial cells. Another study showed that lncRNA GAS5 participates in the renal tubular epithelial fibrosis by regulating miR-96-5p [91]. Our results found that GAS5 can interact with miR-96-5p to target PLC and PKC. The activation of the NF-*κ*B signal can lead to inflammation and vascular complications in T2DM patients. Perhaps, the GAS5/miR-96-5p/PLC-PKC axis is a potential mechanism for the development of diabetic nephropathy, but it still needs a lot of data support. Studies have shown that MIAT mediates high glucose-induced renal tubular epithelial injury [92]. Our investigation predicts that MIAT acts as a sponge for miR-1237-3P, and targeting FN1 leads to a large production of the extracellular matrix. We speculate that the MIAT/miR-1237-3P/FN1 axis may be related to the pathogenesis of diabetic nephropathy, but it needs further research to confirm.

RETRACTED

As far as the current investigation status is concerned, ncRNA is limited to the investigation of the expression level in T2DM. As a response to the lack of investigation on the in-depth mechanism, this study predicts the possible regulatory role of lncRNAs in the diabetic insulin signaling and AGE–RAGE signaling based on bioinformatics, providing a theoretical basis for further investigation.

## 5. Conclusion

This paper summarized the current evidences of the involvement miRNA, lncRNA, and circRNA in the differential expression and interaction with each other in T2DM patients. The interaction between ncRNAs based on the insulin signal and AGE–RAGE signal reveals its important role in insulin resistance and diabetic vascular complications.

## Figures and Tables

**Figure 1:** The flow chart of the data selection and identification process.

**Figure 2:** The pathway enrichment analysis of dysregulated miRNSA targets.

**Figure 3:** Pathway enrichment analysis of dysregulated lncRNA targets.

**Figure 4:** The pathway enrichment analysis of the dysregulated circRNA targets.

**Figure 5:** Noncoding RNA interaction network. CircRNA-lncRNA–miRNA. Triangles represent lncRNA, quadrilaterals represent miRNAs, circles represent cirRNAs, light blues represent predicted miRNAs, red represents high expression levels, and green represents low expression levels.

**Figure 6:** lncRNA-miRNA regulation mechanism diagram based on the insulin signaling pathway.

**Figure 7:** lncRNA-miRNA regulation mechanism diagram based on the AGE-RACE signaling pathway.

**Table 1:** Main features of reports included in the study.

Author, year (ref.)	Country	Sample type	microRNA	Exp change	Assay method	Number of sample (T2DM/NC)	Avg. age (y)	Gender T2DM (M/F)/NC (M/F)	QC
Roux et al., 2018 [15]	France	Plasma	miR-152-3p, miR-196b-5p, miR-362-5p	Up	qRT-PCR	DN (50)/T2DM (50)	T2DM (65.50 ± 8.11)/NC (64.70 ± 7.65)	T2DM(37/13)/NC (37/13)	8
Amr et al., 2018 [16]	Egypt	Plasma	miR-126 and miR-210	Up	qRT-PCR	T2DM (100)/NC (20)	T2DM (56.7 ± 6.9)/NC (58.1 ± 1.1)	T2DM (52/48)/NC (11/9)	7
Ghorbani et al., 2018 [17]	Iran	Serum	miR-21, miR-126, miR-146a	ND	RT-qPCR	T2DM (45)/NC (42)	T2DM (56.5 ± 8.1)/NC (47.6 ± 5.8)	T2DM (26/21)/NC (13/29)	7
Dantas et al., 2018 [18]	Brazil	Plasma	miR-29b and miR-200b	Down	RT-qPCR	T2DM (46)/NC (91)	T2DM (60.0 ± 9.2)/NC (60.3 ± 8.3)	T2DM (47.8%)/NC (33%)	7
Al-Muhtaresh and Al-Kafaji, 2018 [19]	Arabian	Peripheral blood	miR-375 and miR-9	Up	RT-qPCR	T2DM (30)/NC (30)	T2DM (60 ± 12)/NC (56 ± 5.1)	T2DM (12/18)/NC (14/16)	7
Rovira-Llopis et al., 2018 [20]	Spain	Serum	miR-31	Down	RT-qPCR	T2DM(30)/NC(30)	T2DM (61.2 ± 8.4)/NC (56.9 ± 8.7)	T2DM (76.9%)/NC (66.7%)	8
Amr et al., 2018 [16]	Egypt	Plasma	miR126	Down	RT-qPCR	T2DM (30)/NC (30)	T2DM (56.5 ± 7.7)/NC (58.1 ± 1.1)	T2DM (29/25)/NC (11/9)	8
Ding et al., 2017 [21]	China	PBMCs plasma	miR-146a	Down	RT-qPCR	T2DM (30)/NC (30)	T2DM (57 (48–61))/NC (50.5 (45.75–61))	T2DM (11/19)/NC (9/12)	7
de Candia et al., 2017 [22]	Italy	Plasma	miR-122-5p, miR-99a-5p	Up	RT-qPCR	T2DM (9)/NC (9)	T2DM (60.2 ± 8)/NC (57.9 ± 8.9)	T2DM (22%)/NC (44%)	8
			miR-18a-5p, miR-18b-5p, miR-30d-5p	Down					
Yang et al., 2017 [23]	China	Serum	miR-455-5p, miR-454-3p, miR-144-3p, miR-96-5p miR-409-3p	Up	RT-qPCR	T2DM (10)/NC (5)	T2DM (58.2 ± 7.7)/NC (56.4 ± 3.7)	T2DM (2/3)/NC (4/6)	8
			miR-665, miR-766-3p	Down					
Al-Kafaji et al., 2017 [24]	Arabian	Blood	miR-126	Down	RT-qPCR	T2DM (45)/NC (45)	T2DM (61 ± 12)/NC (53 ± 8.6)	T2DM (23/22)/NC (21/24)	7
Ying Shao et al., 2017	China	Serum	microRNA-217	Up	RT-qPCR	T2DM (195)/NC (495)	T2DM (55.96 ± 13.29)/NC (54.12 ± 9.45)	T2DM (255/240)/NC (99/96)	8
Giannella et al., 2017 [25]	Italy	Plasma MP	miR-126-3p	Down	qRT-PCR	T2DM (107)/NC (53)	T2DM (60 ± 1)/NC (57 ± 1)	T2DM (73/34)/NC (30/23)	8
Wang et al., 2017 [26]	China	PBMCs	miR-18a and miR-34c	Up	qRT-PCR	T2DM (117)/NC (105)	T2DM (51.68 ± 8.77)/NC (49.26 ± 9.09)	T2DM (58/47)/NC (68/49)	8
Ma et al., 2017 [27]	China	Serum	miR-3939 and miR-1910-3p	ND	RT-qPCR	DR (45)/T2DM (45)	T2DM (65.42 ± 7.96)/NC (66.24 ± 8.40) DR	NA	6
Wan et al., 2017 [28]	China	Serum	miR-7	Up	qRT-PCR	T2DM (76)/NC (74)	T2DM (48.5 ± 14.5)/NC (48.8 ± 15.2)	T2DM (50% (65.8))/NC (41% (55.4))	8
Jiang et al., 2017 [29]	China	Plasma	miR-21	Up	qRT-PCR	T2DM (189)/NC (115)	T2DM (20–80 y)/NC (48.53 ± 7.26)	T2DM (94/95)/NC (60/55)	9
Zou et al., 2017 [30]	China	Plasma	miR-93	Up	qRT-PCR	T2DM (140)/NC (127)	T2DM (25–72 y)/NC (23–76 y)	T2DM (77/63)/NC (66/61)	8
Shen et al., 2017 [31]	China	PBMCs	miR-125b and miR-34a	Up	qRT-PCR	T2DM (73)/NC (52)	NA	NA	6
Yan et al., 2016 [32]	China	Plasma	miR-1249, miR-320b, miR-6069	Down	qRT-PCR	T2DM (50)/NC (50)	T2DM (46.22 ± 6.897)/NC (45.52 ± 6.215)	T2DM (2/1)/NC (1/2)	7
			miR-572	Up	Microarray	T2DM (3)/NC (3)	T2DM (39.67 ± 1.528)/NC (43.00 ± 10.583)	T2DM (27/23)/NC (22/28)	
Wang et al., 2016 [33]	China	Serum	miR-661, miR-571, miR-770-5p, miR-892b, miR-1303	Up	qRT-PCR	T2DM (92)/NC (92)	T2DM (47.7 ± 13.9)/NC (50.2 ± 14.2)	T2DM (58 (63.0%))/NC (56 (60.9%))	6
Ding et al., 2016 [21]	China	Serum	miR-1183, miR-320c, miR-320d, miR-4530 miR-4534, miR-3960, miR-451a, miR-4443, miR-572	Up	Microarray, qRT-PCR	T2DM (56)/NC (40)	T2DM (58.7 ± 13.5)/NC (63 ± 9.49)	T2DM (27/13)/NC (32/24)	8
Al-Kafaji et al., 2016 [34]	Arabian	Whole blood	miR-126	Down	qRT-PCR	T2DM (50)/NC (52)	T2DM (62.0 ± 10.5)/NC (56 ± 5.2)	T2DM (27/25)/NC (22/28)	8
Al-Kafaji et al., 2016 [24]	Arabian	Whole blood	miR-126	Down	qRT-PCR	T2DM (45)/NC (45)	T2DM (61 ± 12)/NC (53 ± 8.6)	T2DM (23/22)/NC (21/24)	7
Tao et al., 2016 [35]	China	Blood	miR-106b, miR-26a, miR-29b	Up	Microarray, qRT-PCR	T2DM (201)/NC (220)	T2DM (40.7 ± 6.2)/NC (39.2 ± 7.3)	T2DM (36.3%)/NC (41.8%)	8
Ding et al., 2016 [21]	China	Serum	miR-451a, -4534	Up	RT-qPCR	T2DM (40)/NC (56)	61.21	59/37	9
			miR-320d, -3960, -572	Down					
Jansen et al., 2016 [36]	Germany	Plasma	miR-126, -26a	Down	RT-qPCR	T2DM (55)/NC (80)	66.4 ± 10.9	45/90	7
Li et al.,2016 [37]	China	Serum	miR-221/222	Up	RT-qPCR	T2DM (30)/NC (20)	60.28	NA	7
Rezk et al., 2016 [38]	Egypt	Serum	miR-126	Down	RT-qPCR	T2DM (100)/NC (100)	46.95	95/105	9
Seyhan et al., 2016 [39]	USA	Plasma	miR-30d, -34a, -21, -148a	Up	RT-qPCR	T2DM (31)/NC (27)	40.05	30/28	9
Yan et al., 2016 [40]	China	Plasma	miR-572	Up	Microarray RT-qPCR	T2DM (50)/NC (50)	45.87	49/51	8
			miR-1249, -320b	Down					
Wang et al., 2016 [41]	China	Serum	miR-661, -571, -770-5p, -892b, -1303, -15a, -16, -125b, -221, -320a	Up	RT-qPCR	T2DM (92)/NC (92)	48.95	114/70	8
Baldeon et al., 2016	Ecuador	Serum	miR-574-3p, -146a	Down	RT-PCR	T2DM (64)/NC (44)	61 (37–85)	37/71	8
Wang et al., 2016	China	Plasma	miR-296, -9	Down	RT-qPCR	T2DM (150)/NC (150)	48.6 ± 1.7	150/150	7
Long et al., 2015 [42]	China	PBMC	miR-223-3p	Down	RT-qPCR	T2DM (16)/NC (18)	55	20/14	6
Olivieri et al., 2015 [43]	Italy	PBMC	miR-126-3p, -21-5p	Down	RT-qPCR	T2DM (76)/NC (107)	64.79	85/98	9
Higuchi et al., 2015 [44]	Japan	Serum	miR-101, -375, -802	Up	RT-qPCR	T2DM (155)/NC (49)	62.3 ± 13.2	121/83	7
Fluitt et al., 2015 [45]	Bahrain	WB	miRNA-15a	Down	RT-qPCR	T2DM (24)/NC (24)	52 ± 6.0	23/25	8
Lenin et al., 2015	India	PBMC	miR-146a	Down	RT-qPCR	T2DM (35)/NC (35)	47.3 ± 7	36/34	6
Jiao et al., 2015	China	PB	miR-130a, -10b, -143	Down	RT-qPCR	T2DM (30)/NC (42)	56 ± 10	NA	8
Bao et al., 2015	China	Plasma/serum	miR-185	Down	RT-qPCR	T2DM (34)/NC (30)	NA	NA	9
Baldeon et al., 2015	Ecuador	PBMC	miR-34c-5p, -576-3p	Up	Microarray RT-qPCR	T2DM (64)/NC (44)	61 (37–85)	37/71	6
Wu et al., 2015	China	PBMC	miR-21	Up	RT-qPCR	T2DM (18)/NC (18)	53.6 ± 4.6	18/18	7
Ortega et al., 2014 [46]	Spain	Plasma	miR-140-5p, -142-3p, -222	Up	RT-qPCR	T2DM (48)/NC (45)	54 ± 10	93/0	8
			miR-423-5p, -125b, -192, -195, -130b, -532-5p, -126	Down					
Yan et al., 2014	China	Plasma	miR-199a	Up	RT-PCR	T2DM (64)/NC (64)	46–62	NA	8
Lu et al., 2014	China	Plasma	miR-375, miR-126	Up	RT-qPCR	T2DM (30)/NC (30)	53.67 ± 8.92	42/18	8
Wang et al., 2014 [47]	Swedes Iraqis	Plasma	miR-15a, -21, -144, -150, -486-5p	Up	RT-qPCR	T2DM (33)/NC (119)	45–65	83/69	7
			miR-24, -29b, -126, -320a	Down					
Liu et al., 2014 [48]	China	Serum	miR-126	Down	qPCR	T2DM (160)/NC (138)	50.2 ± 6.7	78/82	9
Pan et al., 2014 [49]	China	WB	miR-146a, -155	Down	FQ-PCR	T2DM (36)/NC (32)	61.0 ± 7.0	20/16	9
Yang et al., 2014	China	Serum	miR-23a, let-7i, -486, -96, -186, -191, -192, -146a	Down	RT-qPCR	T2DM (24)/NC (20)	50.60 ± 5.128	(8/16)	9
Santovito et al., 2014 [50]	Germany	Plasma	miR-326	Up	RT-qPCR	T2DM (18)/NC (12)	57.2 ± 9.6	(12/6)	7
			miR-let-7a, let-7f	Down					
Mao et al., 2014	China	Serum	miR-18a	Down	qPCR	T2DM (33)/NC (33)	53.8 (35–72)	13/20	6
Baldeon et al., 2014	Netherlands	Serum	miR-146a	Down	RT-qPCR	T2DM (56)/NC (40)	62 (38–85)	22/34	8
Erener et al., 2014 [51]	China	Plasma	miR-375	Up	qPCR	T2DM (100)/NC (100)	51.33 ± 11.75	54/46	9
Zhang et al., 2014	China	Serum	miR-29b	Up	RT-PCR	T2DM (50)/NC (50)	35–70	30/20	8
Ren et al., 2014	China	Plasma	miR-126	Down	RT-PCR	T2DM (40)/NC (40)	43.0 ± 11.0	24/16	9
Zhou et al., 2013 [52]	China	WB	let-7a	Up	RT-PCR	T2DM (104)/NC (62)	52.8 ± 10.4	59/45	9
Pescador et al., 2013	Spain	Serum	miR-503	Down	RT-qPCR	T2DM (13)/NC (20)	69.40 ± 7.12	(7/6)	8
Zhang et al., 2013 [53]	China	Plasma	miR-126	Down	RT-qPCR	T2DM (30)/NC (30)	63 ± 8.56 (42-73)	16/14	8
Rong et al., 2013 [54]	China	Plasma	miR-146a	Up	qPCR	T2DM (90)/NC (90)	48.50 (42-56)	47/43	9
Corral et al. 2013	Mexico	PBMC	miR-146a, -155	Down	RT-PCR	T2DM (20)/NC (20)	46.2 (35–59)	(11/9)	6
Liang et al., 2010 [55]	China	Serum	miR-29a, -375	Up	RT-FQ-PCR	T2DM (48)/NC (38)	54.9 ± 9.8 (35–72)	27/21	9
Zhou et al., 2012 [56]	China	Serum	miR-181a	Up	RT-PCR	T2DM (20)/NC (20)	NA	NA	7
Meng et al., 2012	China	PBMC	miR-21, -27a, -27b, -126, -130a	Down	Microarray RT-qPCR	T2DM (15)/NC (15)	67 ± 8	(7/8)	8
Karolina et al., 2012 [57]	Singapore	WB	miR-17, -92a, -130a, -195, -197, -509-5p, -652	Down	Microarray RT-qPCR	T2DM (50)/NC (46)	42.02	NA	9
			miR-27a, -150, -192, -320a, -375	Up					
Balasubramanyam et al., 2011 [58]	India	PBMC	miR-146a	Down	RT-qPCR	T2DM (20)/NC (20)	43.7 ± 5.1	NA	8
Caporali et al., 2011	UK	Plasma	miR-503	Up	RT-PCR	T2DM (10)/NC (11)	68.09 ± 9.06	(9/1)	7
		SM	miR-503						
Karolina et al., 2011 [59]	Singapore	WB	miR-15a, -17, -17∗, -23a, -23b, -26a, -26b, -27a, -29b, -29c, -99b∗, -106b, -125a-5p, -125b, -126, -130a, -130b, -142-3p, -151-3p, -151-5p, -183, -185, -190, -193a-3p, -194, -221, -222, -299-3p, -320b, -320c, -320d, -335, -361-3p, -375, -502-3p, -550, -550∗, -589, -620, -629, -665, -886-5p, -1285, -1301	Up	Microarray	T2DM (21)/NC (15)	43.2 (21–70)	21/0	9
			miR-7, -19a, -20a, -20b, -30c, -30e, -34b, -106a, -129-5p, -146b-5p, -185∗, -186, -340, -342-3p, -362-5p, -374b, -519e, -532-3p, -636, -637, -652, -660, -923, -1184, -1297, let-7b∗, let-7d, let-7e, let-7g, let-7i	Down					
			miR-29a, -144, -150, -192, -320a	Up	RT-qPCR				
			miR-30d, -146a, -182	Down					
Kong et al., 2011 [60]	China	Serum	miR-9, -29a, -30d, -34a, -124a, -146a, -375	Up	RT-qPCR	T2DM (18)/NC (19)	47.33 ± 2.617	(9/9)	9
Zampetaki et al., 2010 [61]	UK	Plasma	miR-15a, -20b, -21, -24, -29b, -126, -150, -191, -197, -223, -320, -486	Down	Microarray/RT-qPCR	T2DM (80)/NC (80)	66.3 ± 8.9	30/50	5
			miR-28-3p	Up					
Kong et al., 2010	China	Serum	miR-34a	Up	RT-qPCR	T2DM (18)/NC (26)	47.33 ± 2.62	23/21	

Abbreviations: T2DM: type 2 diabetes; NC: normal control; NA: not available; PB: peripheral blood; PBLC: peripheral blood lymphocytes cell; ND: no difference.

RETRACTED

**Table 2:** Main features of dysregulated lncRNA-related studies in T2DM patients.

Author, year (ref.)	Country	Sample type	lncRNA	Exp change	Assay method	Number of samples	Avg. age (y)	Gender T2DM (M/F)/NC (M/F)	QC
Luo et al., 2018 [62]	China	PBMC	lncRNA MALAT1	Up	Microarray, RT-qPCR	DM (26)/NC (26)	NA	T2DM (F)/NC (0)	7
			lncRNA MEG3	Down					
			lncRNA MALAT1	Up		DPN (26)/NC (26)	NA	NA	
			lncRNA H19, lncRNA PVT1, lncRNA MIR143HG	Down					
Ruan et al., 2018 [63]	China	WB	lncRNA-p3134	Up	Microarray, RT-qPCR	T2DM (30)/NC (30)	(18-65)	NA	6
Wang et al., 2017 [64]	China	WB	lncRNA-n342533, lncRNA-n335556, lncRNA-n336109	Up	Microarray, RT-qPCR	T2DM (60)/NC (60)	T2DM (50.4 ± 13.4)/NC (51.0 ± 9.0)	T2DM (61.7)/NC (58.3)	9
Carter et al., 2015 [65]	USA	Serum	lncRNA GAS5	Down	Microarray, RT-qPCR	T2DM (49)/NC (47)	T2DM (70.3 ± 9.1)/NC (66.9 ± 9.7)	NA	8
de Gonzalo-Calvo et al., 2016 [66]	Spain	Serum	lncRNA-MIAT	Up	RT-qPCR	T2DM (48)/NC (12)	57.6 ± 6.0	M	6
			lncRNA-uc011 mfi.2, lncRNA-uc022bqu.1, lncRNA-uc022bqw.1	Down					
Mansoori et al., 2018 [67]	Iran	PBMC	LINC00523, LINC00994	Down	RT-qPCR	T2DM (100)/NC (100)	59.50 ± 1.08	T2DM (36/64)	8
Li et al., 2017 [68]	China	WB	LncRNA ENST00000550337.1, LncRNA-uc011llp.1, LncRNA-uc011fnr.2	Down	Microarray	T2DM (6)/NC (6)	T2DM (62.3 ± 6.2)/NC (60 ± 2.3)	T2DM (1/1)	8
					RT-qPCR	T2DM (80)/NC (84)	T2DM (50 ± 6.0)/NC (49.3 ± 5.1)	T2DM (11/9)	
Qiong Yin et al., 2017 [69]	China	Plasma	lncRNA GAS5	Down	RT-qPCR	T2DM (10)/NC (30)	41 ± 9.8	T2DM (4/6)	8
Yu et al., 2017 [70]	China	Serum	LncRNA NONRATT021972	Up	RT-qPCR	T2DM (154)/NC (154)	55–65	T2DM (M)	8

Abbreviations: T2DM: type 2 diabetes; NC: normal control; NA: not available; PB: peripheral blood; PBLC: peripheral blood lymphocytes cell.

**Table 3:** Main features of dysregulated circRNA-related studies in T2DM patients.

Author, year (ref.)	Country	Sample type	circRNA	Exp change	Assay method	Number of samples	Avg. age (y)	Gender (M/F) NC	QC
Fang et al., 2018 [14]	China	PBLC	circANKRD36	Up	RT-PCR	T2DM (43)/NC (45)	T2DM (65.2 ± 13.23)/NC (66.2 ± 5.49)	M/F = 2/3	8
Li et al., 2017 [71]	China	PB	circRNA11806-28, circRNA6510-1, circRNA11783-2	Down	Microarray	T2DM (6)/NC (6)	T2DM (62.3 ± 6.2)/NC (60 ± 2.3)	M/F = 1/1	8
					RT-qPCR	T2DM (80)/NC (84)	T2DM (50.6 ± 5.7)/NC (49.0 ± 5.5)	64/100	
Gu et al., 2017 [72]	China	Serum	circRNA-063981, circRNA_404457, circ-RNA_100750, circRNA_406918, circRNA_104387, circRNA_103410, circRNA_100192	Up	Microarray	T2DMR (5)/NC (5)	T2DM (67.40 ± 13.92)/NC (60.60 ± 12.82)	M/F = 2/3	8
					qRT-PCR	T2DMR (14)/NC (16)	NA	NA	
Zhao et al., 2017 [73]	China	PB	circRNA_0054633, circRNA_0068087	Up	qRT-PCR, microarray	T2DM (64)/NC (60)	T2DM (32 cases ≥ 50, 32 cases < 50)/NC (23 cases ≥ 5, 37 cases < 50)	M/F = 64/60	8
Zhang et al., 2017 [74]	China	Plasma	circRNA_0005015	Up	qRT-PCR	T2DMr (20)/NC (20)	NA	NA	6

Abbreviations: T2DM: type 2 diabetes; NC: normal control; NA: not available; PB, peripheral blood; PBLC, peripheral blood lymphocytes cell.

RETRACTED

## Data Availability

The data of differentially expressed noncoding RNAs in type 2 diabetes patients were acquired from PubMed, MiRWalk, and other databases; please visit https://pubmed.ncbi.nlm.nih.gov/, http://zmf.umm.uni-heidelberg.de/apps/zmf/mirwalk2/, https://circinteractome.nia.nih.gov

## Supplementary Materials

Supplementary Materials Supplementary Figure 1. The red squares in the pathway represent genes that are regulated by lncRNA in patients with T2DM. Construction of a network based on the KEGG pathway map: AGE–RAGE signaling pathway in diabetic complications (KEGG hsa04933).  Figure 3(a), Insulin signaling pathway (KEGG hsa04910). Figures 3(b) and 3(c), Insulin resistance (hsa04931). Supplementary Figure 2. The red squares in the pathway represent genes that are regulated by lncRNA in patients with T2DM. Construction of a network based on the KEGG pathway map: AGE–RAGE signaling pathway in diabetic complications (KEGG hsa04933).  Figure 4(a), Insulin signaling pathway (KEGG hsa04910). Figures 4(b) and 4(c), Insulin resistance (KEGG hsa04931). Supplementary Figure 3. 3a shows the interaction network of lncRNA and miRNA; 3b shows the interaction network of circRNA and miRNA.
